The article "Comparison of Different Therapeutic Effects of T-MIST for Chronic Idiopathic Tinnitus" was published in 2022. Journal: Biomed Res Int.

# Comparison of Different Therapeutic Effects of T-MIST for Chronic Idiopathic Tinnitus

**DOI:** 10.1155/2022/9236822

**Published:** 2022-09-29

**Authors:** Chaoqun Liang, Qi Fang, Hongjun Chen, Zhixian Wang, Jianming Yang

**Affiliations:** Department of Otorhinolaryngology, Head and Neck Surgery, The Second Affiliated Hospital of Anhui Medical University, Hefei, Anhui, China

## Abstract

**Objective:**

Tinnitus, as a common clinical symptom, has the characteristics of high incidence and great heterogeneity among different patients. As one of the common treatment strategies for tinnitus, this study is aimed at exploring the factors influencing tinnitus sound therapy and the correlation between different tinnitus acoustic characteristics.

**Methods:**

315 patients with chronic tinnitus were enrolled and divided into three groups according to the tinnitus multielement integration sound therapy (T-MIST): (1) vanishing, (2) remission, and (3) unchanged. The general characteristics, psychoacoustic scores (tinnitus handicap inventory (THI) and visual analog scale (VAS)), residual inhibition (RI), degree of hearing loss, and tinnitus characteristics of each group were compared. Finally, we analyze the predictive significance of different features for acoustic effects.

**Results:**

The frequency of tinnitus in the vanishing group was higher than that in the remission and unchanged groups (*P* < 0.05). There were no differences in age, initial onset time, course of the disease, and VSAD between the vanishing group and the unchanged group (*P* > 0.05). High-frequency tinnitus may predict the vanishing of tinnitus after treatment (*P* < 0.05), but the degree of hearing loss, tinnitus characteristics (loudness and frequency), and psychoacoustic score (THI and VAS) were only weakly correlated (*P* < 0.05). Residual inhibition test (RI) was an independent risk factor for the efficacy of acoustic therapy (*P* < 0.001).

**Conclusion:**

The patients were divided into three groups by T-MIST treatment effect; Kruskal-Wallis test and chi-square test were used to compare the baseline information of each group. Then, we analyzed the correlation between patient characteristics and psychoacoustic scores. Finally, logistic regression was performed to explore predictors that might influence the treatment effect. High-frequency tinnitus may have a better therapeutic effect; age, disease course, and other factors can not be stable explanation factors for a poor therapeutic effect of tinnitus. The residual inhibition (RI) test was an independent factor in predicting the efficacy of T-MIST.

## 1. Introduction

Idiopathic tinnitus is the perception of sound in the absence of auditory stimulation, often accompanied by hearing loss, which can cause psychological changes in patients, resulting in anxiety, depression, and other manifestations [1, 2]. Tinnitus occurs in about 10% to 25% of adults [3, 4] which had become a widespread public health burden. Due to the development of neuroimaging in recent years, it is currently believed that auditory impairment can cause neural synchronization [5, 6] and plasticity changes [7, 8]. The reorganization of various neural networks such as temporal lobe emotion, auditory nerve, and limbic system is also thought to be the neural source of tinnitus. Neuroimaging studies have identified abnormal connections involving the auditory, affective, thalamic, and somatosensory systems in the brains of tinnitus patients [9–12]. As one of the main treatment methods for tinnitus, sound therapy is based on the theory that it is through auditory stimulation to reverse the abnormal nerve excitation and brain area connection, to alleviate or eliminate tinnitus [13–15]. Tinnitus multielement integration sound therapy (T-MIST) is an acoustic therapy for tinnitus using full precision audiometry (FPT) to match frequency and loudness for tinnitus patients, combined with background noise and soothing music [16]. So far, we have not found literature comparing the treatment effects of different groups. The purpose of this study was to investigate the basic characteristics of patients with different T-MIST efficacy and the indicators that might indicate the efficacy of acoustic therapy.

## 2. Methods

### 2.1. Participants

A total of 315 tinnitus patients aged 18 to 81 years were included in this study. These patients were admitted to the Otorhinolaryngology Department of the Second Affiliated Hospital of Anhui Medical University from June 2018 to August 2020. These patients were divided into three groups based on the efficacy of T-MIST: vanishing, remission, and unchanged. All participants had to have subjective tinnitus for at least 3 months. Based on the patient's history, symptoms, and detailed ontological examinations (otoscopy, audiology, and computed tomography), all diseases of the middle and inner ears that may cause tinnitus such as otitis media, Meniere's disease, auditory neuropathy, and sudden hearing loss were excluded. Patients with cardiovascular and cerebrovascular diseases, systemic metabolic and immune diseases, and malignant tumor history were excluded as well. All participants verbally agreed to use their medical data. This study was supported by the Ethics Committee of the Second Affiliated Hospital of Anhui Medical University: YJ-YX2019-039.

### 2.2. Evaluation

All patients were evaluated by the tinnitus handicap inventory (THI) [17] and the visual analog scale (VAS) [18] before and after sound therapy. THI included 25 functional questions about tinnitus emotions and disasters, each offering three options: “no,” “sometimes,” and “always” with a score of “0,” “2,” and “4” for each option. VAS assesses the distress of tinnitus patients in two aspects: (1) how loud is your tinnitus and (2) how stressful is your tinnitus. The VAS score ranges from 0 (no tinnitus/no pressure) to 10 (very loud tinnitus/high pressure). The severity of tinnitus and improvement of tinnitus disturbance were evaluated according to THI and VAS scores before and after treatment.

### 2.3. Hearing Measurement

Considering that there may be patients with “hidden hearing loss” [19], all the patients included in the study were subjected to full precision hearing measurement to determine the hearing threshold. When the patients' full frequency hearing was less than 25 dBHL, they were considered to have no hearing loss. According to WHO's hearing classification standard, the mean hearing thresholds of patients at 500 kHz, 1000 kHz, and 2000 kHz were calculated. Tinnitus matching (frequency and loudness), residual inhibition test, and T-MIST were also completed on the tinnitus comprehensive rehabilitation therapy pairing platform (Foshan Primus Medical Technology Co., Ltd. Sftest330). The device complies with GB/T-16403 standards. All patients were examined and treated by the same audiologist.

### 2.4. Tinnitus Match

Tinnitus frequency matching was performed on the side of patients with severe tinnitus. Based on FPT, three similar frequency test sounds were sent to the patients. After the patients selected the frequency with a similar tinnitus frequency, three adjacent test sounds were sent again with the selected frequency sound as the center. This is repeated until the patient determines that the test tone is the tinnitus frequency tone, thus determining the tinnitus loudness. Based on tinnitus frequency matching, the test soundness was gradually increased based on 1 dB in tinnitus frequency. The loudness was determined as tinnitus loudness when a patient could not feel the presence of tinnitus [20].

### 2.5. Residual Inhibition Test

Based on tinnitus frequency and loudness, the patients were given a narrow-band noise stimulation sound 10 dB louder than tinnitus, which lasted for 1 min, and subjective tinnitus sensation was recorded after stimulation. According to the classification of patients' feelings, the results of the residual inhibition test were divided into three levels: completely positive means that the patient's tinnitus has completely disappeared, partially positive means that the tinnitus loudness or frequency has improved, and negative means that the patient's tinnitus has no change [21].

### 2.6. Tinnitus Multielement Integration Sound Therapy (T-MIST)

The T-MIST was the combination of three sounds: i-tone, dual-sound, and Transfocus. (1) The i-tone has fine frequency selection characteristics and is mainly used to match the frequency of tinnitus to achieve suppression and regulation of tinnitus at specific frequencies. Loudness corresponds to tinnitus loudness. (2) The dual-sound has specific frequency characteristics, dynamic range, and psychoperceptual properties. It mainly uses its specific frequency to act on the tinnitus frequency to establish a new sound perception, covering the sound perception of tinnitus, which contains a variety of natural environment sounds. (3) Transfocus can create a pleasant and relaxing psychological perception; it has psychological perception properties, frequency-free properties, and various types of music. Patients can choose the desired two-tone and Transfocus type and comfortable loudness. The playing time is 15 min each time [16]. According to patients' subjective feelings after treatment, the treatment results can be divided into (1) vanishing, (2) remission, and (3) unchanged. Due to the development of neuroimaging, more and more studies have proved that there are abnormal links between the auditory system, emotional system, thalamic system, and somatosensory system in patients with tinnitus [9–11, 22, 23]. Sound stimulation reduces spontaneous activity in the primary auditory cortex in tinnitus patients. Improves tinnitus perception by reversing abnormal activity in primary auditory cortex neurons and a broad network of frontal, parietal, and limbic regions [16, 24–26].

### 2.7. Statistical Analysis

All data were statistically analyzed by IBM SPSS Statistics 26. Descriptive data are expressed as median (interquartile range) or ratio (as appropriate). Kolmogorov-Smirnov was used for normality analysis of grouped data. Levene's test was used to evaluate whether each group had homogeneity of variance, and the rank test was used for continuous data. The chi-square test was used for counting data. Pairwise comparison was performed for variables with statistically significant differences among multiple groups, and *P* values were adjusted. ROC curve was used to determine the prognostic critical value, and Spearman correlation analysis was used to analyze the correlation between nonnormal data and grade data. Univariate logistic regression and multivariate logistic regression were performed to explore independent risk factors.

## 3. Results

### 3.1. Comparison between Groups of T-MIST

Basic information for comparison between the three groups is shown in Table 1. There were statistically significant differences in age (*P* = 0.008), initial onset time (*P* = 0.020), course of disease (*P* = 0.007), VASD (*P* = 0.035), frequency of tinnitus (*P* = 0.016), and residual inhibition test (*P* < 0.001) among the three groups.

### 3.2. Post Hoc Comparisons and ROC Curves

(1) There were statistically significant differences in age (*P* = 0.006), initial onset time (*P* = 0.018), disease duration (*P* = 0.010), VASD (*P* = 0.043), and residual inhibition test (*P* < 0.001) between the remission group and the unchanged group, but there was no significant difference in tinnitus frequency between the two groups (Figures 1(a)–1(e)). (2) Since it was observed that the frequency of tinnitus in the vanishing group was significantly higher than that in the other two groups, we performed a ROC curve to evaluate the diagnostic efficacy of tinnitus frequency on acoustic therapy. The results indicated that the area under the tinnitus frequency curve was 0.637 (95% CI, 0.548-0.726, *P* = 0.004) (Figure 1(f)).

### 3.3. Correlation Analysis of Tinnitus Characteristics

Spearman correlation analysis is used to explore the correlation between tinnitus and psychoacoustics. The correlation between RI and T-MIST was rs = 0.464 and *P* < 0.001, and the correlation between VASB and THIB was rs = 0.661 and *P* < 0.001. The correlations of hearing loss, tinnitus loudness, and frequency with VASB and THIB were rs = 0.257 and *P* < 0.001, rs = 0.270 and *P* < 0.001, rs = 0.194 and *P* = 0.001, rs = 0.215 and *P* < 0.001, rs = −0.158 and *P* = 0.005, and rs = −0.111 and *P* = 0.049, respectively (Table 2).

### 3.4. Risk Factors of T-MIST Treatment Outcome

According to the outcome of T-MIST treatment, age, initial onset time, tinnitus course, VASD, and residual inhibition test were included in the logistic regression. The results showed that the parallel line test failed and multiclassification logistic regression was used instead. After adjusting for risk factors for all important outcomes, residual inhibition test results remained an independent predictor of T-MIST therapeutic efficacy, with adjusted OR (vanishing/unchanged) of 0.071 (95% CI, 0.035-0.143, *P* < 0.001) and OR (remission/unchanged) of 0.399 (95% CI, 0.259-0.614, *P* < 0.001) (Table 3).

## 4. Discussion

Due to the heterogeneity of tinnitus etiology and the difficulty of treatment, many attempts have been made to treat tinnitus. As a form of tinnitus treatment, T-MIST has been analyzed in the literature on its therapeutic effect, but the predictors of its treatment are inconclusive. The purpose of this study is to explore whether tinnitus patients with different T-MIST treatment effects have different clinical characteristics and provide help for the follow-up T-MIST treatment. Although there are differences in the incidence of tinnitus in different genders and different sides of tinnitus [4], we have not found any difference in the therapeutic effect of tinnitus sound between the two groups. What is puzzling is that there is no significant difference in tinnitus loudness, average hearing threshold, THIB, VASB, and THID among the three groups, which is contrary to our traditional cognition [27]. In general, we think that tinnitus loudness and average hearing threshold can further affect the therapeutic effect by affecting the psychology of patients [28, 29]. In our study, hearing loss and tinnitus characteristics (loudness and frequency) were indeed positively correlated with the psychoacoustic score of tinnitus, but their correlation was small, which also demonstrated its limitations in predicting psychoacoustic outcomes in tinnitus patients. The significantly higher frequency of tinnitus in the vanishing group than in the remission and unchanged groups may be explained by the fact that the daily auditory frequency in humans is predominantly low to medium frequencies, thus making it easier to benefit from transient neural suppression with sound therapy [30]. At the same time, when the ROC analysis was carried out, the results showed that the tinnitus frequency was helpful to the outcome of T-MIST. For indicators such as age, initial onset time, tinnitus course, and VASD, except for VASD, which was lowest in the unchanged group, the rest of the indicators were lower in the remission group, while there was no obvious difference between the vanishing group and the unchanged group. The occurrence of this phenomenon may be related to the self-adaptation of tinnitus patients [31]. There were significant differences in pairwise comparison among the three groups of RI, and the correlation analysis between RI and T-MIST showed a moderate correlation, which was the same as the previous scholars' conclusion [32]. At the same time, in the multiple logistic regression model, we found that only RI was an independent positive predictor of T-MIST treatment, which complements the gaps in previous studies. Similar to the fact that hearing loss is not directly related to tinnitus, we did not find the possibility of compensating sound to affect the outcome of T-MIST treatment [33]. Due to the limitation of sample information included in this study, it is not possible to analyze the prognostic effects of cardiovascular, lipid metabolism, endocrine and other systemic diseases, and ear concomitant symptoms such as vertigo on the prognosis of sound therapy.

## 5. Conclusion

T-MIST is a simple treatment without significant side effects; this study demonstrates that patients with high-frequency tinnitus can get better results in T-MIST treatment, consistent with a negative correlation between frequency and tinnitus psychoacoustics. RI can provide an independent prediction for tinnitus treatment. Traditional psychoacoustic indicators such as THI and VAS cannot predict the therapeutic effect. Tinnitus loudness and hearing loss had little correlation with tinnitus annoyance degree and did not affect the treatment results of tinnitus. Finally, this study does not support age as a stable prognostic factor for tinnitus acoustic therapy.

## Figures and Tables

**Figure 1:** Post hoc comparison results among the groups and the frequency ROC curve.

**Table 1:** Basic information for comparison between the T-MIST groups (*N* = 315)^∗^.

	Vanishing	Remission	Unchanged	*P*
Number	42	146	127	
Gender (male/female)	23/19	79/67	75/52	0.699
Age (years)	44.00 (28.75-59.25)	41.50 (28.75-51.00)	48.00 (34.00-55.00)	0.008
Initial onset time (years)	42.54 (22.85-53.67)	38.00 (25.72-49.08)	43.00 (31.50-52.83)	0.020
Left ear/right ear/both ears	8/13/21	56/34/56	39/35/53	0.200
Hearing loss: yes/no	12/30	46/100	36/91	0.835
Course of disease (years)	1.00 (0.50-5.50)	1.00 (0.50-3.00)	2.00 (1.00-5.00)	0.007
THIB	45.00 (25.5-57.00)	40.00 (28.00-40.00)	44.00 (28.00-62.00)	0.855
THIA	33.00 (18.00-42.75)	30.50 (18.00-50.25)	32.00 (16.00-50.00)	0.343
VASB	5.00 (4.00-7.00)	5.00 (4.00-7.00)	5.00 (4.00-7.00)	0.535
VASA	3.00 (2.00-5.00)	4.00 (2.00-5.00)	4.00 (3.00-6.00)	0.107
THID	8.00 (0.00-20.25)	8.00 (2.00-15.00)	4.00 (0.00-13.00)	0.095
VASD	1.00 (0.00-3.00)	1.00 (0.00-2.00)	0.00 (0.00-2.00)	0.035
Tinnitus loudness (dB)	39.00 (20.00-59.50)	43.00 (22.00-58.00)	46.00 (24.00-64.00)	0.181
Tinnitus frequency (Hz)	5047 (4000-7663)	4000 (1260-6082)	3775.00 (1260-5993)	0.016
Average threshold of hearing (dB)	20.00 (14.58-30.00)	18.33 (13.33-31.67)	21.67 (15.00-35.00)	0.136
RI: completely/partially/negative	23/16/3	11/75/60	6/31/90	<0.001

^∗^The values are given as median with its interquartile range (25–75th). The values are given as the number of cases. THIB, THIA, VASB, VASA, THID, VASD: THI before treatment, THI after treatment, VAS before treatment, VAS after treatment, THIB-THIA, VASB-VASA; average threshold of hearing: average hearing thresholds of 500 kHz, 1000 kHz, and 2000 kHz; RI: residual inhibition test.

**Table 2:** Correlation analysis of tinnitus characteristics.

Factor A	Factor B	*r*_*s*_	*P*
T-MIST	RI	0.464	<0.001

VASB	THIB	0.661	<0.001

Average threshold of hearing	VASB	0.257	<0.001
	THIB	0.270	<0.001

Tinnitus loudness (dB)	VASB	0.194	0.001
	THIB	0.215	<0.001

Tinnitus frequency (Hz)	VASB	-0.158	0.005
	THIB	-0.111	0.049

RI: residual inhibition test; THIB, THIA, VASB, VASA, THID, VASD: THI before treatment, THI after treatment, VAS before treatment, VAS after treatment, THIB-THIA, VASB-VASA; average threshold of hearing: average hearing thresholds of 500 kHz, 1000 kHz, and 2000 kHz.

**Table 3:** Potential factors associated with T-MIST.

	Univariate analysis		Multivariate analysis	
	Vanishing/unchanged	Remission/unchanged	Vanishing/unchanged	Remission/unchanged
	OR (95% CI)	OR (95% CI)	OR (95% CI)	OR (95% CI)
Predictor				
Age (years)	0.995 (0.971-1.019)	0.975 (0.958-0.991)	0.996 (0.967-1.026)	0.975 (0.958-0.993)
Initial onset time (years)	0.996 (0.972-1.020)	0.977 (0.961-0.994)		
Course of disease (years)	0.991 (0.917-1.071)	0.976 (0.925-1.031)		
Gender (male)	1.191 (0.590-2.407)	1.223 (0.756-1.978)		
Left ear (both)	0.518 (0.208-1.290)	1.359 (0.780-2.368)		
Right ear (both)	0.937 (0.416-2.113)	0.919 (0.503-1.681)		
Hearing loss (no)	0.989 (0.457-2.142)	0.860 (0.511-1.447)		
THIB	1.000 (0.985-1.016)	0.997 (0.987-1.008)		
THIA	0.995 (0.979-1.011)	0.997 (0.986-1.008)		
VASB	0.988 (0.835-1.170)	0.949 (0.845-1.066)		
VASA	0.881 (0.749-1.036)	0.992 (0.829-1.026)		
THID	1.018 (0.993-1.045)	1.001 (0.981-1.021)		
VASD	1.212 (1.000-1.470)	1.074 (0.927-1.244)		
Tinnitus loudness (dB)	0.991 (0.976-1.007)	0.990 (0.980-1.001)		
Tinnitus frequency (<4623.5 Hz)	3.435 (1.631-7.235)	1.169 (0.721-1.896)	2.853 (1.185-6.874)	1.027 (0.613-1.721)
Average hearing (dB)	0.727 (0.499-1.059)	0.809 (0.646-1.013)		
RI	0.063 (0.031-0.127)	0.394 (0.257-0.604)	0.071 (0.035-0.143)	0.399 (0.259-0.614)

Vanishing, remission, unchanged: the treatment results of T-MIST; THIB, THIA, VASB, VASA, THID, VASD: THI before treatment, THI after treatment, VAS before treatment, VAS after treatment, THIB-THID, VASB-VASD; average hearing: average hearing thresholds of 500 kHz, 1000 kHz, and 2000 kHz; RI: residual inhibition test.

## Data Availability

The data for this article can be obtained from corresponding authors where reasonable.
